This article has been retracted.

# Antenatal Steroid Therapy for Fetal Lung Maturation and the Subsequent Risk of Childhood Asthma: A Longitudinal Analysis

**DOI:** 10.1155/2010/789748

**Published:** 2010-06-15

**Authors:** Jason D. Pole, Cameron A. Mustard, Teresa To, Joseph Beyene, Alexander C. Allen

**Affiliations:** ^1^Dalla Lana School of Public Health, University of Toronto, Toronto, ON, Canada M5T 3M7; ^2^Pediatric Oncology Group of Ontario, Toronto, ON, Canada M5G 1V2; ^3^Child Health Evaluative Sciences, The Hospital for Sick Children, Toronto, ON, Canada M5G 1X8; ^4^Department of Clinical Epidemiology & Biostatistics, McMaster University, Hamilton, ON, Canada L8N 3Z5; ^5^Perinatal Epidemiology Research Unit, Departments of Obstetrics and Gynecology and Pediatrics, Dalhousie University, Halifax, Nova Scotia, Canada B3K 6R8

## Abstract

This study was designed to test the hypothesis that fetal exposure to corticosteroids in the antenatal period is an independent risk factor for the development of asthma in early childhood with little or no effect in later childhood. A population-based cohort study of all pregnant women who resided in Nova Scotia, Canada, and gave birth to a singleton fetus between 1989 and 1998 was undertaken. After a priori specified exclusions, 80,448 infants were available for analysis. Using linked health care utilization records, incident asthma cases developed after 36 months of age were identified. Extended Cox proportional hazards models were used to estimate hazard ratios while controlling for confounders. Exposure to corticosteroids during pregnancy was associated with a risk of asthma in childhood between 3–5 years of age: adjusted hazard ratio of 1.19 (95% confidence interval: 1.03, 1.39), with no association noted after 5 years of age: adjusted hazard ratio for 5–7 years was 1.06 (95% confidence interval: 0.86, 1.30) and for 8 or greater years was 0.74 (95% confidence interval: 0.54, 1.03). Antenatal steroid therapy appears to be an independent risk factor for the development of asthma between 3 and 5 years of age.

## 1. Introduction

Research on the etiology and natural history of asthma has identified a web of predisposing factors (e.g., genetics, atopy), causal factors that may sensitize the airways (e.g., animal dander, dust mites, workplace allergens) and contributing factors (perinatal events such as mode of delivery, exposure to cigarette smoke during pregnancy, gestational age and childhood respiratory infections, air quality, socioeconomic status, and pollution) [1–6]. Conclusions that can be drawn from this research outline a myriad of exposures and complex interactions in the etiology of pediatric asthma [7–10].

Given the complex nature of pediatric asthma etiology, factors in the perinatal period that would predispose individuals to asthma are of particular interest [11, 12]. Corticosteroid (CS) therapy, administered during labour and delivery to accelerate fetal lung maturation, has not been fully examined as a potential risk factor for the development of asthma in humans [13]. CS therapy has been shown to alter the development of the fetal lung and has been linked, in animal studies, to changes in brain chemistry and subsequent hypertension later in life [14–28]. Complex time-dependent relationships between CS therapy and subsequent lung function in animals has been noted [29].

The use of CS therapy, in Canada, among preterm infants before 34 weeks' gestation has increased in the last 15 years from less than 25 percent to approximately 60 percent [30, 31]. This increase of CS therapy follows from randomized controlled trial evidence indicating increased infant survival among preterm infants exposed to antenatal CS therapy [32].

A limited number of previous studies have investigated lung function (not asthma) in childhood among those previously exposed to CS therapy [33–36]. The small sample sizes and convenience samples of these studies do not provide sufficient evidence for or against an association between CS therapy and asthma [13]. Therefore, a large population-based cohort study where confounding by indication can be controlled is warranted.

This study was designed to test the hypothesis that fetal exposure to corticosteroids in the antenatal period is an independent risk factor for the development of asthma in childhood. Further, the risk of asthma is hypothesized to be greater in the early childhood years and attenuated in later childhood.

## 2. Methods

A population-based cohort study of all pregnant women who resided in Nova Scotia, Canada and gave birth to a singleton fetus between January 1, 1989, and December 31, 1998, and lived to discharge was undertaken.

Data from The Maternal-Child Health Database (MCHD) were used. The MCHD is a longitudinal population-based database of all mothers and infants delivered while resident in Nova Scotia that is linked to health services utilization data. Four independently collected linked databases comprise the MCHD used in this study including data from the Nova Scotia Atlee Perinatal Database (NSAPD), the Nova Scotia physician visits Medical Services Insurance File database, the Nova Scotia Vital Statistics Database and the Nova Scotia portion of the Canadian Institute for Health Information hospital admissions database.

Pregnancies that resulted in the birth of more than one infant (twins, triplets, quadruplets) differ from singleton pregnancies both physiologically and obstetrically and therefore were not eligible for inclusion. Mothers who suffer from thyroid conditions (due to higher levels of hormones already present) and mothers experiencing active asthma during the gestational period (due to increased risk of obstetrical complications and the possibility of fetal exposure to steroids because of the pharmaceutical interventions used to manage the mothers asthma) were also excluded [37–39].

Previous work in Canada has established that health service administrative records can be used to identify and describe children with asthma [40–43]. The definition of asthma employed in this study was based on this previous work, determined by examining physician visits or hospitalizations where the primary diagnostic field was for asthma or asthma-like conditions (asthma: ICD-9-CM code 493, bronchitis: ICD-9-CM code 490, or bronchiolitis: ICD-9-CM code 466). Subjects who experienced at least two health care interactions in any 365 day period, starting at 156 weeks post birth (3 years), where the diagnosis was asthma or an asthma-like condition and at least one visit was not in the winter period (December to March inclusive), or experienced one hospitalization specifically for asthma (ICD-9-CM code 493) were considered to be asthmatic [40]. This definition captures all levels of asthma severity.

A second more conservative definition of asthma was developed to examine the potential that the primary definition would be too encompassing and therefore have a high level of misclassification. The conservative definition of asthma was similar to the primary definition except that only interactions where asthma (ICD-CM code 493) was the primary diagnostic field were considered.

The primary exposure of interest is antenatal CS therapy. Maternal systemic steroid therapy is coded in the NSAPD [44]. The first dose of the first course of betamethasone or dexamethasone coupled with the timing of the administration is recorded. For this study, infants were considered exposed to CS therapy if either of these drugs was administered regardless of timing.

Numerous potential risk factors for childhood asthma have been identified in the literature. Potential confounders considered in this analysis included the infant's sex, gestational age at birth, maternal age, one minute Apgar score, administration of surfactant, infant's birth weight, delivery by caesarian section, maternal smoking during the gestational period, socio-economic status (SES), hyaline membrane disease, bronchopulmonary dysplasia, maternal insulin dependant diabetes mellitus, gestational diabetes, number of siblings, and year of birth.

The infant's gestational age at birth, in completed weeks, was examined both continuously and as a dichotomous variable indicating full term/preterm, with full term being 37 or more completed weeks of gestation. Infants born at an early gestational age are at increased risk of poor lung function and preterm labour is often used as an indication for CS therapy [30, 45–47]. 

### 2.1. Confounding

Control for confounding by indication was achieved in this study given not all infants who are preterm or low birth weight were exposed to CS therapy and a portion of infants who are full-term or full birth weight will have been exposed. There is a portion of infants in each year of the cohort where the therapy is clinically indicated, but for various reasons not administered (e.g., where mothers presented to the hospital too late). Also, there is a portion of infants in each year of the cohort where the therapy is clinically indicated and administered, but for various reasons delivery was able to be delayed until the infant was delivered full term. Therefore, each year a proportion of preterm and low birth weight infants are unexposed and a portion of full-term infants are exposed to CS therapy allowing for differences in the development of childhood asthma to be examined.

Maternal age was examined continuously. Given maternal age has been shown to be related to preterm birth and related to obstetrical complications leading to the administration of CS, maternal age was only considered as a confounder in this analysis [31, 48]. The infants one minute Apgar score (examined in three categories, 0–3, 4–6, 7–10) has been shown to be an independent risk factor for childhood asthma [49]. Delivery by caesarean section was examined as a dichotomous variable where, regardless of other obstetrical interventions during delivery (e.g., the use of forceps prior to surgery), if the infant was ultimately born by caesarean section it was considered a caesarean section. Delivery by caesarean section is related to CS therapy and CS therapy has been shown to be associated with poor lung function in the infant [49, 50]. Maternal smoking during pregnancy was examined as a dichotomous variable. Cigarette exposure during the gestational period has been shown to be related to the development of childhood asthma and risk of obstetrical complications (including prematurity) that are related to the administration of CS [47, 51–56]. Differences in the complication rate and the potential for threatened preterm labour is increased when the mother is diagnosed with either type 1 diabetes mellitus or gestational diabetes.

Hyaline membrane disease is a respiratory condition in the infant that is often associated with preterm delivery and subsequent morbidity. CS therapy was primarily instituted to ameliorate this disease. However, the administration of surfactant to alleviate various respiratory difficulties in the infant after birth, such as hyaline membrane disease, has been shown to be related to both long term lung function and the use of CS therapy [57–60].

Due to the declining incidence of asthma over the time period under study, the year of birth was used to control for birth cohort effects (temporal effects).

A greater number of older siblings in a household has been shown to be associated with reduced risk of childhood asthma and forms part of the basis for the hygiene hypothesis [61–63]. Also related to the hygiene hypothesis is the socioeconomic status of the infants family [64, 65]. Mothers who are of low socioeconomic status are also more likely to have various pregnancy complications that include threatened preterm labour [66]. Therefore, two socioeconomic status measures were used in this study. Marital status at the time of delivery (married or common law versus single, widowed, divorced, or separated) and quintiles of neighbourhood income (based on the postal code of residence at the time of delivery).

### 2.2. Analysis

Extended Cox proportional hazards regression models were used to analyse the data [67]. Time zero was recorded as the date of birth. Duration of follow-up was measured in weeks. Subjects were censored the week they were identified as having asthma, died or were lost to follow-up. Given the outcome of asthma was not considered before 156 weeks the minimum amount of follow-up time required to be included in this analysis was therefore 156 weeks. 

A Cox proportional hazards regression stratified by antenatal steroid therapy was utilized to assess the time dependant hazard comparing subjects that received and did not receive steroid therapy. A kernel smoothing method was utilized to remove the extreme variability in the time-specific hazard estimates [68, 69].

Given that one mother may give birth to more than one infant in the cohort an examination of robust variance estimates was undertaken using a sandwich estimator. The nonindependence altered the variance estimates by less than 5 percent so no consideration of this nonindependence was given in subsequent analysis.

To quantitatively assess if the hazard ratio for the association between exposure to antenatal corticosteroids and the subsequent development of asthma changes with time, an extended Cox proportional hazards regression with time-dependant covariates was used. The effect of steroid administration through time was described by three hazard ratios; one when time was between 156 and 260 weeks, one when time was between 261 and 364 weeks and one when time was greater than 364 weeks. These time periods were selected based on an examination of the smoothed figure derived from the stratified Cox model.

All potential confounders were examined with nested models with the time-dependant covariates for steroid administration. Each potential confounder's effect on the parameter estimates for antenatal steroid therapy (early, mid and late) was assessed by examining the percentage difference in the parameter estimates from a model with and without the potential confounder. Differences larger than 10 percent in any one of the parameter estimates was considered evidence of confounding [70]. Potential cofounders that did not demonstrate evidence of confounding were not retained in the final models.

Thus, the statistical model for the final analysis was as follows:

(1) $$\begin{array}{cc} & h\left(t,X\left(t\right)\right)=h_{0}\left(t\right)\exp\;[\beta_{1}\left(\text{steroid}\right)g_{1}\left(t\right)+\beta_{2}\left(\text{steroid}\right)g_{2}\left(t\right)\;\\ & \;\;\;\;\;\;\;\;\;\;+\beta_{3}\left(\text{steroid}\right)g_{3}\left(t\right)+\beta_{x}], \end{array}$$

where

(2) $$\begin{array}{cc} g_{1}\left(t\right) & =\{\begin{array}{cc} 1 & \text{if}\;\;\;\;156<t\leq 260\;\;\;\text{weeks},\\ 0 & \text{if}\;\;\;\;t<260\;\;\;\text{weeks}, \end{array}\\ g_{2}\left(t\right) & =\{\begin{array}{cc} 1 & \text{if}\;\;\;\;261\leq t\leq 364\;\;\;\text{weeks},\\ 0 & \text{if}\;\;\;\;t<261\;\;\text{or}\;\;\;t>364\;\;\;\text{weeks}, \end{array}\;\\ g_{3}\left(t\right) & =\{\begin{array}{cc} 1, & \text{if}\;\;\;\;t\geq 365\;\;\;\text{weeks},\\ 0, & \text{if}\;\;\;\;t<365\;\;\;\text{weeks}, \end{array}\;\\ \beta_{x} & =\{\begin{array}{c} x\;\;\;\text{other}\;\text{covariates}.\; \end{array} \end{array}$$

  

 All statistical analyses were performed using SAS version 8.2.

## 3. Results

There were a total of 113,145 births between January 1, 1989, and December 31, 1998, in Nova Scotia. Exclusions included 1,325 fetal, neonatal or infant deaths that occurred before 1 year of age, 2,408 infants who were delivered from a multiple gestation, 4,958 infants who were born to mothers experiencing active asthma during the gestational period and a further 89 infants were excluded because they were born to mothers experiencing endocrine abnormalities.

There were 104,365 infants eligible for record linkage. Birth records for 18,627 infants could not be successfully linked to the health care follow-up data due to errors or missing information with the provincial unique identifier. Due to deaths, migration, and other events an additional 3,484 infants did not have 156 or more weeks of follow-up time. A further 1,671 infants did not have either a birth weight or gestational age recorded (which is required for the analysis), 135 infants were greater than or less than three standard deviations from their mean sex-specific birth weight for gestational age and therefore were excluded. This left 80,448 infants for analysis.

Table 1 provides descriptive statistics for the study sample by asthma status. Both a row and column percentage is provided to assist in the interpretation of the relationships. The asthma incidence among birth cohorts peaked in 1989 and has been on a decline since. The number of siblings, income, marital status, mean birth weight, mean gestational age and mean maternal age at birth are similar between asthmatics and nonasthmatics. Infants born preterm had an elevated incidence of asthma over the follow-up period. As expected, children who developed asthma had higher prevalence of caesarean section, surfactant administration, maternal smoking, hyaline membrane disease and bronchopulmonary dysplasia compared to children who did not develop asthma. The median overall follow-up time was nearly 8.5 years (440 weeks). On average asthma developed in this cohort at approximately 5.5 years of age (287 weeks).

Table 2 provides the rates of antenatal steroid therapy administration and preterm birth by year of birth. The use of antenatal steroid therapy increased 3-fold over the 10-year time period of the study, from a rate of 7.5 in 1989 to 23.7 per 1,000 births in 1998. The preterm birth rate increased approximately 30 percent over the same period, from a rate of 40.5 in 1989 to 52.7 per 1,000 live births in 1998.

Figure 1 provides the smoothed adjusted hazard function over time, stratified by antenatal steroid therapy. Adjustments were made for the infant's sex, gestational age at birth and year of birth. Given the smoothing algorithm used a bandwidth of 75 weeks, the tales of the curves have not been estimated. The figure provides evidence that the hazard for developing asthma differs by antenatal steroid therapy dependant on time. The difference is greatest in the early period, diminishing over the middle period with little differences noted beyond 7 years (400 weeks).

Table 3 contains the estimated adjusted hazard ratios for the development of asthma for antenatal steroid therapy from 3 to 5, 6 to 7 and 8, or greater years of age along with the estimates for all other confounders in the model. Adjustments were made for infant's sex, gestational age at birth and an indicator for perterm birth, one minute Apgar score, administration of surfactant, infant's birth weight, delivery by caesarian section, maternal smoking during the gestational period, hyaline membrane disease, bronchopulmonary dysplasia, number of siblings and year of birth. Unadjusted hazard ratio estimates are also provided for the antenatal steroid exposure. The effect of antenatal steroid therapy on the development of asthma is seen to be larger in early childhood (HR = 1.19, 95% CI: 1.03, 1.39) with no effect noted in mid childhood (HR = 1.06, 95% CI: 0.86, 1.30) and potentially a protective effect in late childhood (HR = 0.74, 95% CI: 0.54, 1.03).

When considering the more conservative definition of asthma the prevalence of asthma dropped from 25.4% to 18.0%. The estimated adjusted hazard ratios for the development of asthma for antenatal steroid therapy from 3 to 5, 6 to 7 and 8 or greater years of age were HR = 1.37 (95% CI: 1.15, 1.62), HR = 1.17 (95% CI: 0.93, 1.49) and HR = 0.92 (95% CI: 0.67, 1.26), respectively. Adjustments were made for the same confounders as in the main model.

## 4. Discussion

Antenatal steroid therapy appears to be an independent risk factor for the development of childhood asthma after controlling for confounding. The risk appears to be time-dependent with the highest risk early in childhood and diminishing as the child ages. The reasons for this increase risk are not obvious but many animal studies have established latent effects of corticosteroid exposure in utero. 

Although a mechanistic link between antenatal corticosteroid therapy and the onset of asthma in childhood has not been fully established [71], wide ranging effects of corticosteroid therapy have been demonstrated. The alteration in brain chemistry and hypothalamic-pituitary-adrenal (HPA) axis, the shift in immune function and other wide-ranging latent effects such as changes in kidney development and subsequent hypertension all provide biological plausibility for a link to childhood asthma. 

Time-dependent complications associated with antenatal corticosteroid therapy have been demonstrated [15, 16]. Corticosteroids have been shown to affect HPA development in primates, sheep and to a limited extent in humans [17–20]. The HPA axis is important in regulating the physical growth and organ development of the neonate [18]. The timing of exposure to corticosteroids within a species, late in gestation, has been shown by Matthews to be critical with regard to the effect on the HPA axis [17, 21]. Published and unpublished work by Clifton in Australia indicates that corticosteroid exposure not only alters the HPA axis but also influences the Th1/Th2 ratio in favour of Th2 [72].

Strengths of this study are rooted in the large population cohort that were assembled and followed for extended lengths of time. The availability of potential confounders for control was extensive. Control for confounding by indication was also inherent in this study design providing considerable methodological strength.

The retrospective nature of this study design has a number of limitations. The reliability and validity of an asthma diagnosis in the MSI data is unknown. Errors in the primary reason for admission in the CIHI Hospital Discharge Data may occur when several competing causes of admission are present in any one individual. Errors of this sort, with both databases, would have a conservative effect on the estimate of association generated in this study. 

When considering the more conservative definition of asthma the pattern of early childhood risk for the development of asthma after antenatal exposure to corticosteroids remains the same as with the main asthma definition. As expected with this definition the risk estimate, particularly in the early childhood period is greater. This sensitivity analysis lends credence to the hazard ratio estimates using the main asthma definition.

Limitations in the measure of exposure exist, in that there is no measure of the CS that crosses the placenta and is biologically available to each fetus. Information that pertains to multiple exposure to CS therapy and the actual amount of medication administered is not recorded in the NSAPD. With all data limitations outlined, bias would only result if there was a systematic difference between those exposed to CS therapy and those not exposed. There is no indication that physician billing or hospital discharge records would be different based on exposure.

Given that this study is focussed on mothers and infants from the province of Nova Scotia, Canada, any findings from this current study would need to be replicated in other populations to strengthen external validity. Although no factors specifically related to the biological effects of CS therapy are postulated to differ between this population and others, other factors related to childhood asthma may differ. The trend in asthma incidence by birth year for this population appears to be different than that of other populations and therefore replication of these findings in different populations is warranted.

Continued research into the perinatal factors in the etiology of childhood asthma is warranted. Information continues to surface that draws attention to the potential long term consequences of exposures *in utero* and subsequent disease risk. Cohort studies that examine the time-dependant effects are crucial in establishing periods of disease susceptibility. Although only a small, but significant, elevated risk for childhood asthma and antenatal steroid exposure was demonstrated in the current study, further research into the smallest possible dose required for the steroid to achieve the desired post-natal effect could be undertaken potentially limiting the long term consequences such as childhood asthma.

## Figures and Tables

**Figure 1:** Smoothed Hazard Function Estimates by Antenatal Steroid Therapy. Note: Adjusted for gender, gestational age and year of birth.

**Table 1:** Descriptive characteristics of the study sample by asthma status.

	Asthma							
	No			Yes			Total	
		%			%			
	Num	Row	Column	Num	Row	Column	Num	%*
Total	59,975	74.6	100.0	20,473	25.4	100.0	80,448	100.0

Birth year								
1989	3,823	65.1	6.4	2,051	34.9	10.0	5,874	7.3
1990	5,816	66.5	9.7	2,931	33.5	14.3	8,747	10.9
1991	5,671	67.2	9.5	2,773	32.8	13.5	8,444	10.5
1992	6,020	71.7	10.0	2,374	28.3	11.6	8,394	10.4
1993	6,135	74.0	10.2	2,152	26.0	10.5	8,287	10.3
1994	6,524	75.9	10.9	2,067	24.1	10.1	8,591	10.7
1995	6,503	77.4	10.8	1,896	22.6	9.3	8,399	10.4
1996	6,793	80.7	11.3	1,629	19.3	8.0	8,422	10.5
1997	6,465	81.8	10.8	1,440	18.2	7.0	7,905	9.8
1998	6,225	84.3	10.4	1,160	15.7	5.7	7,385	9.2

Antenatal steroid exposure	773	68.1	1.3	362	31.9	1.8	1,135	1.4

Number of siblings								
0	25,916	72.2	43.2	9,972	27.8	48.7	35,888	44.6
1	21,753	75.1	36.3	7,199	24.9	35.2	28,952	36.0
2	8,691	78.1	14.5	2,435	21.9	11.9	11,126	13.8
3+	3,608	80.7	6.0	864	19.3	4.2	4,472	5.6

Preterm birth (<37 weeks)	2,534	68.1	4.2	1,189	31.9	5.8	3,723	4.6

Caesarean section	10,873	71.9	18.1	4,253	28.1	20.8	15,126	18.8

Income								
Quintile 1	12,693	73.6	21.5	4,547	26.4	22.7	17,240	21.4
Quintile 2	12,619	74.3	21.4	4,359	25.7	21.7	16,978	21.1
Quintile 3	11,368	75.2	19.3	3,749	24.8	18.7	15,117	18.8
Quintile 4	12,435	74.6	21.1	4,235	25.4	21.1	16,670	20.7
Quintile 5	9,873	75.7	16.7	3,174	24.3	15.8	13,047	16.2

Surfactant administration	139	59.9	0.2	93	40.1	0.5	232	0.3

1 Minute Apgar score								
0–3	1,309	70.4	2.2	550	29.6	2.7	1,859	2.3
4–6	4,375	71.9	7.3	1,712	28.1	8.4	6,087	7.6
7–10	54,070	74.9	90.5	18,137	25.1	88.9	72,207	89.8

Maternal smoking	16,421	72.6	27.4	6,211	27.4	30.3	22,632	28.1
Married/Common law	42,671	74.6	71.1	14,566	25.4	71.1	57,237	71.1
Hyaline membrane disease	672	62.3	1.1	406	37.7	2.0	1,078	1.3
Bronchopulmonary dysplasia	97	54.2	0.2	82	45.8	0.4	179	0.2
Duration: weeks (mean, SD)	512.3	155.3		287.2	116.6		455.0	176.2
Birth weight: grams (mean, SD)	3,487.4	554.7		3,444.3	592.1		3,476.5	564.7
Gestational age: weeks (mean, SD)	39.5	1.7		39.3	1.9		39.4	1.7
Maternal age: years (mean, SD)	26.7	5.3		26.4	5.2		26.6	5.3

Note: All totals do not add to grand total given missing values for some variables.

*Percent of total cohort.

**Table 2:** Rates of antenatal steroid therapy administration and preterm birth by year of birth.

	Total births	Steroid administration					
		Preterm		Full term		Preterm birth	
	Num	Num	Rate	Num	Rate	Num	Rate
Year of birth							
1989	5,874	26	109.24	18	3.19	238	40.52
1990	8,747	49	129.63	18	2.15	378	43.21
1991	8,444	58	164.31	28	3.46	353	41.80
1992	8,394	79	201.02	40	5.00	393	46.82
1993	8,287	69	195.47	36	4.54	353	42.60
1994	8,591	68	181.82	48	5.84	374	43.53
1995	8,399	78	186.16	34	4.26	419	49.89
1996	8,422	99	235.71	46	5.75	420	49.87
1997	7,905	106	261.08	60	8.00	406	51.36
1998	7,385	99	254.50	76	10.86	389	52.67

Total	80,448	731	196.35	404	5.27	3,723	46.28

Note: Rate is per 1,000 births.

**Table 3:** Association between antenatal steroid therapy exposure and childhood asthma.

	Adjusted		Unadjusted	
	HR	95% CI	HR	95% CI
Antenatal steroid exposure				
3–5 years	1.19	1.03–1.39	1.55	1.36–1.77
6–7 years	1.06	0.86–1.30	1.36	1.12–1.65
8+ years	0.74	0.54–1.03	0.98	0.72–1.34

Male gender	1.24	1.21–1.28	—	
Preterm birth (<37 weeks)	1.03	0.95–1.12	—	

Number of siblings				
0	1.00	—		
1	0.90	0.88–0.93	—	
2	0.78	0.74–0.82	—	
3+	0.67	0.62–0.72	—	

Bronchopulmonary Dysplasia	0.98	0.74–1.31	—	
Hyaline Membrane Disease	1.14	1.01–1.30	—	
Surfactant Administration	1.07	0.82–1.40	—	

1 Minute Apgar Score				
0–3	1.00	—		
4–6	0.95	0.86–1.05	—	
7–10	0.87	0.79–0.95	—	

Caesarean section	1.11	1.07–1.15	—	
Maternal smoking	1.12	1.09–1.16	—	
Birth weight (per 500 grams)	1.00	0.98–1.01	—	
Gestational age (weeks)	0.97	0.96–0.98	—	

Birth year				
1989	1.47	1.37–1.59		
1990	1.45	1.35–1.56	—	
1991	1.49	1.39–1.60	—	
1992	1.28	1.19–1.37	—	
1993	1.21	1.12–1.30	—	
1994	1.14	1.06–1.23	—	
1995	1.12	1.04–1.20	—	
1996	0.99	0.92–1.07	—	
1997	1.02	0.95–1.11	—	
1998	1.00	—		

Note: Adjustment for all other confounders in table.
